# Identification of novel signaling components in N,N’-Dinitrosopiperazine-mediated metastasis of nasopharyngeal Carcinoma by quantitative phosphoproteomics

This article has been retracted.

**DOI:** 10.1186/1471-2407-14-243

**Published:** 2014-04-05

**Authors:** Damao Huang, Yuejin Li, Na Liu, Zhenlin Zhang, Zhengke Peng, Chaojun Duan, Xiaowei Tang, Gongjun Tan, Guangrong Yan, Faqing Tang

**Affiliations:** 1 Medical Research Center and Clinical Laboratory, Xiangya Hospital, Central South University, Changsha 410008, Hunan, China; 2 Clinical Laboratory and Medical Research Center, Zhuhai Hospital, Jinan University, Zhuhai 519000, Guangdong, China; 3 Metallurgical Science and Engineering, Central South University, Changsha 410008, PR China; 4 Institute of Life and Health Engineering, and National Engineering and Research Center for Genetic Medicine, Jinan University, Guangzhou 510632, China

**Keywords:** Dinitrosopiperazine, Nasopharyngeal carcinoma, Metastasis, Quantitative phosphoproteomics

## Abstract

**Background:**

Nasopharyngeal carcinoma (NPC) is a highly invasive and metastatic cancer. N,N’*-*dinitrosopiperazine (DNP), a carcinogen with specificity for nasopharyngeal epithelium, facilitates NPC metastasis. However, the underlying mechanism is not known.

**Methods:**

Quantitative phosphoproteomics, using stable isotope labeling of amino acids in cell cultures, was employed to identify phosphoproteins associated with NPC metastasis mediated by DNP. NPC cell line 6-10B, which is relatively less metastatic, was used to investigate DNP-mediated metastasis. Boyden chamber invasion assay was used to measure DNP-induced motility and invasion, and nude mice were used to verify DNP-mediated metastasis in vivo. Several different phosphoproteins detected by proteomics analysis were verified by immunoblotting. DNP-mediated metastasis facilitated by lysine-rich CEACAM1 co-isolated protein (LYRIC) phosphorylation at serine 568 was confirmed using mutations targeting the phosphorylation site of LYRIC. DNP-mediated metastasis through LYRIC phosphorylation was confirmed in the NPC cell line CNE1. DNP-mediated LYRIC phosphorylation at serine 568 was also verified in metastatic tumors of BABL/c nude mice.

**Results:**

Boyden chamber invasion assay indicated that DNP mediated cell motility and invasion of NPC cell 6-10B in vitro*,* and experiments with nude mice indicated that DNP increased 6-10B metastasis in vivo. In the phosphoproteomics analysis, we detected 216 phosphorylation sites on 130 proteins; among these, 48 phosphorylation sites on 30 unique phosphopeptides were modulated by DNP by at least 1.5-fold. DNP mediated the expression of phosphorylated GTPase, ferritin, LYRIC, and RNA polymerase, and it decreased the expression of phosphorylated torsin-1A protein 1. Furthermore, DNP induced LYRIC phosphorylation at serine 568 to facilitate cell motility and invasion, whereas DNP-mediated motility and invasion was decreased when serine 568 in LYRIC was mutated. In another NPC cell line, CNE1, DNP also mediated cell motility and invasion followed by enhanced phosphorylation of LYRIC at serine 568. Finally, phosphorylated-LYRIC expression at serine 568 was significantly increased in metastatic tumors induced by DNP.

**Conclusion:**

DNP regulates multiple signaling pathways through protein phosphorylation, including the phosphorylation of LYRIC at serine 568, and mediates NPC metastasis. These findings provide insights on the complexity and dynamics of DNP-facilitated metastasis, and may help to gain a better understanding of the mechanisms by clarifying NPC-induced metastasis.

## Background

Nasopharyngeal carcinoma (NPC) is endemic in certain regions of the world, particularly in Southeast Asia, with an annual incidence of 30–80 per 100,000 people in southern China [1]. NPC has invasive and metastatic features, and approximately 90% of patients show cervical lymph node metastasis at the time of initial diagnosis [2]. Therapeutic limitations in advanced NPC have resulted in high rates of both local recurrence and distant metastasis [3-5]. However, the underlying mechanism that favors this high metastasis is not clearly understood.

Protein phosphorylation is an important molecular event related to signaling pathways that control various biological responses. Phosphorylation can affect the function of a protein in many ways by increasing or decreasing its activity, mediating translocation between subcellular compartments, initiating/disrupting protein–protein interactions, or affecting their stabilization in signaling pathways [6]. Protein phosphorylation and dephosphorylation are regulated by the balanced activity of protein kinases and phosphatases. Kinase-mediated phosphorylation plays an important role in controlling signaling pathways [7,8]. In carcinogenesis, carcinogens may facilitate constitutive activation of some protein kinases such as Rho-kinase, protein kinase C (PKC), epithelial growth factor receptor, Bcr-Abl, and ErbB-2 [9-11]. The hyperactivation of some protein kinases has been associated with tumor metastasis [12]. In NPC, the carcinogen N,N’*-*Dinitrosopiperazine (DNP) has been reported to activate Rho-kinase and PKC and promote NPC metastasis [13].

In Chinese populations, the relative risk of NPC associated with those consume salt-preserved fish on a weekly or daily basis, compared with those who do not consume salt-preserved fish, was generally in the range 1.4–3.2 and 1.8–7.5, respectively [14-19]. Consumption of salted fish is an important source of nitrosamines. Some bacteria can also induce the conversion of nitrates into nitrites, forming important carcinogenic N-nitroso compounds [20]. DNP is a predominant volatile nitrosamine in salted fish [18,21,22]. DNP not only induces NPC [21,23], but also facilitates NPC metastasis [13,24]. In clinical assays, NPC patients with lymph node metastasis have a higher level of serum DNP than that in non-metastatic patients [13]. Experimental studies indicate that DNP activates Rho-kinase and PKC, mediates ezrin phosphorylation, induces motility and invasion of cells, and promotes tumor metastasis [13]. As a carcinogen for NPC, DNP may also induce the expression of other phosphorylated proteins and activate multiple signaling pathways that are involved in NPC metastasis. To clarify DNP-mediated phosphorylation and associated signaling pathways, and to identify novel signaling targets of DNP, we employed a proteomics approach to comprehensively identify DNP-regulated phosphoproteins and phosphosites by using high-resolution mass spectrometry (MS) in combination with TiO_2_ phosphopeptide enrichment and stable isotope labeling of amino acids in cell culture (SILAC). Thirty phosphoproteins were found to be regulated by DNP, most of which have not been previously reported to be involved in NPC metastasis. Analysis of this critical information helps us better understand the complex mechanism by which DNP regulates cancer the growth and proliferation of cancer cells. Many novel signaling molecules in DNP-regulated signaling pathways have been identified here for the first time, including lysine-rich CEACAM1 co-isolated protein (LYRIC) phosphorylation at serine 568.

## Methods

### Reagents and antibodies

DNP was a kind gift from the Cancer Research Institute, Central South University (Hunan, China), and its chemical structure is shown in Figure 1A. Chemical reagents, including Tris–HCl, sodium dodecyl sulfate (SDS), Na_2_S_2_O_3_, K_3_Fe (CN)_6_, l-1-tosylamide-2-phenylethyl chloromethyl ketone-treated trypsin, ethylene diamine tetraacetic acid (EDTA), NH_4_HCO_3_, acrylamide, urea, thiourea, NP-40, Triton-X100, DL-dithiothreitol (DTT), phenylmethane-sulfonyl-fluoride (PMSF), 3-[(3-cholamidopropyl) dimethylammonio]-1-propanesulfonate, and pharmolyte, were purchased from Sigma-Aldrich (St. Louis, MO). Lactate dehydrogenase (LDH) assay reagents were purchased from Autec Diagnostica Co (Botzing, Germany). The antibody against Rho GTPase was purchased from Cell Signaling Technology (Danvers, MA), and antibodies against ferritin, RNA polymerase, and serine were purchased from Santa Cruz Biotechnology, Inc. (Santa Cruz, CA). Torsin-1A protein 1 antibody was purchased from Abcam (Cambridge, UK), and antibody to LYRIC was purchased from Biocompare. The phospho-antibody against LYRIC serine 568 was purchased from Abcam. The secondary antibodies, horseradish peroxidase-linked anti-mouse immunoglobulin G and anti-rabbit immunoglobulin G, were purchased from Santa Cruz Biotechnology, Inc. Immunoblotting detection reagents, glutathione-sepharose 4B, and the BCA protein assay kit were purchased from Amersham Biosciences (Buckinghamshire, UK). Dimethyl sulfoxide (DMSO) and 3-(4,5-dimethylthiazol-2-yl)-5-(3-carboxymethoxyphenyl)-2-(4-ulfophenyl)-2H-tetrazolium (MTT) were purchased from Sigma-Aldrich. The QuikChange II Site-Directed Mutagenesis Kit was purchased from Amersham Pharmacia Biotech (Piscataway, NJ).

**Figure 1:** **Non-cytotoxic concentration of N,N’-dinitrosopiperazine (DNP) on the labeled 6-10B cells. A**, Structure of DNP, an N-nitroso compound. **B**, The labeled 6-10B cells were treated with 0.5, 1, 2, 4, 6, 8, 10, 20, 40, 80, or 100 μM DNP for 48 h before being subjected to MTT cell viability assay. The inhibitory rates of DNP were calculated to the labeled 6-10B. **C**, After 6-10B cells were treated with 2, 4, 6, 8, 10, or 20 μM DNP for 48 h, the media were subjected to LDH assay. OD indicates the relative optical density at 563 nm. The data indicate the LDH activity per 1 L media. Data are presented as means ± SD from 3 independent experiments, and statistically analyzed using the Student’s *t-* test (*, p < 0.05).

### Cell culture and SILAC labeling

Human NPC cell line 6-10B was purchased from State Key Laboratory of Oncology in South China (Guangzhou, China); human NPC cell line CNE1 was a kind gift from the Cancer Research Institute, Central South University (Hunan, China). These two cell lines have a low metastatic ability [25]. The 6-10B cells were grown in Dulbecco’s modified Eagle medium containing “light” (^12^C_6_) or “heavy” (^13^C_6_) lysine supplemented with dialyzed fetal bovine serum at 37°C for 2 weeks. At about 30% confluence, the “heavy” labeled 6-10B cells were treated with 6 µΜ DNP for 48 h after the labeled amino acids in cell populations were identified as being completely incorporated, following a previously established protocol [26]. The “light” labeled 6-10B cells were treated with only DMSO. The cells were then harvested and suspended with lysis buffer (50 mM Tris–HCl pH 8.0, 1 mM EDTA, 2% SDS, 1 mM DTT, 10 mM PMSF, 1 mM NaF, 1 mM Na_3_VO_4_, and protease inhibitor cocktail). The lysate was centrifuged at 13,200 rpm at 4°C for 30 min. The supernatant fractions were collected, and protein concentration was determined by BCA assay (Pierce, Rockford, IL).

### MTT assay

To determine the non-cytotoxic concentration of DNP, MTT assay was performed to determine cell viability [27]. In brief, the labeled 6-10B cells were seeded in 96-well plates at a density of 3.5 × 10^3^ cells/well and treated with 0 to ~100 μM DNP for 48 h at 37°C. For DNP treatment, the DNP crystals were dissolved in DMSO, and appropriate amounts of DNP stock solution were added to the cultured cells to achieve the indicated concentrations. The cells were then incubated for the indicated times. After the exposure period, the media were removed, and the cells were washed with phosphate-buffered saline (PBS). Then, the media were changed, and cells were incubated with 100 μL MTT (5 mg/mL) per well for 4 h. The number of viable cells per dish was directly proportional to the production and detection of formazan crystals, which was solubilized in isopropanol and measured spectrophotometrically at 563 nm. The inhibitory rates of DNP were calculated for the labeled 6-10B cells.

### Lactose dehydrogenase (LDH) assay

To further confirm the non-cytotoxic concentration of DNP to the labeled 6-10B cells, the LDH activity in cell culture media was determined after DNP treatment. Briefly, the cells were seeded in 6-well plates at a density of 2 × 10^4^ cells/well and treated with 0–10 μM DNP for 24 h at 37°C. After the exposure period, the media were collected for measurement of LDH activity using the LDH assay kit (Autec Diagnostica, Freiberg, Germany)

### Cell motility and invasion assay

For cell invasion assay, the labeled 6-10B cells were treated with the indicated concentrations of DNP for the indicated times. After DNP treatment, the cells were removed by trypsinization, and their invasiveness was tested using Boyden chamber invasion assay in vitro [28]. Matrigel (Collaborative Biomedical Products, Bedford, MA) was diluted to 25 mg/50 mL with cold-filtered distilled water and applied to 8-mm pore size polycarbonate membrane filters. Treated cells were seeded in the upper part of Boyden chamber (NeuroProbe, Cabin John, MD) at a density of 1.5 × 10^4^ cells/well in 50 μL of serum-free-medium and then incubated for 12 h at 37°C. The bottom chamber also contained standard medium with 20% fetal bovine serum. The cells invading to the lower surface of the membrane were fixed with methanol and stained with hematoxylin and eosin. Random fields were counted to determine the number of invading cells under a light microscope. To determine cell motility, the cells were seeded in Boyden Chamber on membrane filters that were not coated with Matrigel. Cellular migration was measured as described in the motility assay [28]. Statistical analysis was performed, corrected with cell viability, to clarify the effect of DNP.

### Animals

Twenty female nude BABL/c mice (approximately 5–6 weeks old) were purchased from the Animal Center of Central South University. They were maintained under laminar airflow conditions in the Laboratory for Experiments, Central South University. The studies were conducted according to the standards established by the Guidelines for Care and Use of Laboratory Animals of Central South University.

### Evaluation of the effect of DNP on NPC metastasis in nude mice

The metastatic effect of DNP on labeled 6-10B cells was determined in vivo as described previously with some modifications [29]. In brief, 100-μL aliquots of labeled 6-10B cell suspensions (1 × 10^4^ cells) with or without DNP treatment were mixed with Matrigel and then respectively injected into the tail veins of nude mice (10 mice per group). Metastasis was assessed by observing metastasized nodes in lungs on day 30 post-injection. The present study protocols were approved by the ethical committees at Zhuhai Hospital of Jinan University and Xiangya Hospital of Central South University.

### Protein digestion in solution

The proteins were digested in solution as previously described [30] with minor modifications. The “heavy” and “light” labeled proteins were mixed at a ratio of 1:1 by protein weight, and 2 mg of the mixed proteins was reduced at 37°C for 3 h in 10 mM DTT and subsequently alkylated in the dark with 20 mM iodoacetamide at room temperature for 1 h. The proteins were precipitated in ice-cold buffer (50% acetone, 50% ethanol, 0.1% HAc). The precipitated proteins were resuspended in 100 mM NH_4_HCO_3_, and initially digested with trypsin (1:50, w/w) at 37°C for 4 h. Further digestion was carried out by adding trypsin (1:50, w/w) and incubating overnight at 37°C. The digests were evaporated to about 20 μL in a SpeedVac centrifuge for phosphopeptide enrichment.

### Phosphopeptide enrichment using TiO_2_

Phosphopeptide enrichment was carried out following the manufacture’s instructions provided with the Proteoextract phosphopeptide enrichment TiO_2_ kit (Calbiochem, Gibbstown, NJ). In brief, trypsin-digested samples (2 mg mixed proteins) were diluted at the ratio of 1:4 with TiO_2_ Phosphobind Buffer containing 2,5-dihydroxybenzoic acid to achieve a final volume of 200 μL. The diluted peptide mixtures were mixed with TiO_2_ Phosphobind Resin and then incubated for 10 min at room temperature. The TiO_2_ Phosphobind Resin was washed twice, once with Wash Buffer 1 and once with Wash Buffer 2 from the kit. Finally, the phosphopeptides were eluted twice from the TiO_2_ Phosphobind Resin using the Elution Buffer supplied in the kit. The collected phosphopeptide solutions were evaporated to dryness in a SpeedVac centrifuge and used for liquid chromatography tandem MS (LC–MS/MS) analysis.

### Strong-cation exchange (SCX)-LC–MS/MS analysis

An xA linear ion trap/Orbitrap (LTQ-Orbitrap) hybrid mass spectrometer (Thermo Electron, Bremen, Germany) coupled with strong-cation exchange (SCX) and nano-reverse-phase LC (Thermo Electron, Bremen, Germany) was used to analyze the enriched phosphopeptides as previously described [31] with minor modifications. In brief, the phosphopeptides were first loaded onto an SCX column (0.8 × 50 mm, Zorbax Bio-SCX Series II; Agilent Technology) by using an autosampler with a flow rate of 10 μL/min, eluted with different concentrations (0, 5, 10, 40, 80, and 200 mM, and 1 M) of NH_4_Cl, and loaded onto a C18 reverse-phase column (150 × 0.075 mm, Zorbax 300SB-C18, 3.5 μm, Agilent Technology) with a flow rate of 300 nL/min for 150 min. The peptide mixtures were further eluted with a 0–40% gradient of Buffer A (0.1% formic acid, and 5% acetonitrile) to Buffer B (0.1% formic acid and 95% acetonitrile), and mass of the peptides were then detected using an LTQ-Orbitrap mass spectrometer. This analysis was performed in a data-dependent mode in which acquisitions were automatically switched between MS and MS/MS. In each cycle, a full MS scan was carried out in the Orbitrap, followed by 5 MS/MS scans for 5 most intense ions in the LTQ. When an ion had a neutral loss peak at −98.00, −58.00, −49.00, −38.67, −32.67, and −24.50 Da in MS/MS scan and was one of the 5 most intense ions in MS/MS spectrum, the ion was further selected for an MS/MS/MS scan. The neutral loss peaks at 98.00, 49.00, 32.67 and 24.50 Da indicate the losses of phosphate groups in peptides with 1, 2, 3, and 4 charge states, respectively, in the MS scan, while the 58.00 and 38.67 Da peaks indicate the loss of a phosphate group and a H_2_O in peptides with 2 and 3 charge states, respectively, in the MS/MS scan.

### Phosphopeptide identification and quantitation, and phosphosite validation

The mass list of the peaks was generated in the Mascot generic format using DTASuperCharge V 1.31 (SourceForge) for database search, and the derived peak lists were searched using the Mascot 2.2.04 search engine (Matrix Science, London, UK) against real and decoy IPI human databases (V3.56) containing 76,539 human protein entries. The following search criteria were employed: full tryptic specificity was required, 2 missed cleavages were allowed, and carbamidomethylation was set as a fixed modification, whereas oxidation (M), phospho (ST), and phospho (Y) were considered variable modifications. Precursor ion mass tolerances and fragment ion mass tolerances were 10 ppm and 0.5 Da, respectively. Mass spectra of identified phosphopeptides with peptide scores >10 were further processed and validated with the MSQuant 1.5 software for post-translational modification (PTM) score analysis and quantitation, with default settings [32]. The SILAC ratio normalization was automatically processed by MSQuant 1.5 software. The relative standard deviation (RSD) of peptide quantitation was calculated as previously described [31]. In brief, the RSD of peptide phosphorylation was determined by using average SD of all quantified peptide counts of a unique phosphopeptide in 2 biological replicates, i.e., it was calculated using the total SD/counts of the unique phosphopeptide. The SD of unique phosphopeptide in a hit was automatically generated by the MSQuant program. All the spectra of these potential and decoy phosphopeptides were confirmed by manual interpretation of MS/MS ion spectra using the criteria described previously [32,33]. Briefly, 5 filters for peptide identification were applied as follows: (1) the peptide score threshold was 10; (2) the PTM score threshold was 14; (3) all phosphorylated serine (p-Ser) and phosphorylated threonine (p-Thr) peptides were required to show a pronounced neutral loss of phosphoric acid from the precursor ion and/or fragment ions, or to trigger the neutral loss-dependent MS/MS/MS scan; (4) at least 3 consecutive b- and/or y-ion series were required; and (5) the sum of peptide and PTM scores was greater than 31. Other parameters were those included in the default settings. The estimated false positive rate based on the decoy database search was 1.0%. For ambiguous phosphosites, the probabilities for phosphorylation at each site were calculated based on PTM scores as previously described [34]. Phosphorylation sites with localization probabilities >0.75 were reported as class I phosphosites, and localization probabilities between 0.75 and 0.25 were considered to be class II sites. Phosphorylation sites with a localization probability <0.25 were discarded.

### Immunoblotting analysis

Cellular extracts were prepared as described previously [27]. After DNP treatment, the cell samples were disrupted with 0.6 mL lysis buffer. The cell lysates were then subjected to centrifugation at 10000 × *g* for 10 min at 4°C. The resultant protein concentration of each sample was determined using BCA Protein Assay (Bio-Rad Laboratories, Inc., Hercules, CA). Forty micrograms protein from each sample was separated on 10% or 12% polyacrylamide gel and transferred onto a nitrocellulose membrane. The blot was subsequently incubated with 5% non-fat milk in PBS for 1 h to block non-specific binding and incubated with Rho GTPase, ferritin, RNA polymerase, Torsin-1A, or LYRIC antibody for 2 h, and then with an appropriate peroxidase-conjugated secondary antibody for 1 h. All incubations were carried out at 37°C, and the membranes were washed with PBS after the incubations. Finally, the membrane was washed with PBS three times, and the signal was developed using 4-chloro-1-naphthol/3,3-*O*-diaminobenzidine, and the relative photographic density was quantitated by a gel documentation and analysis system. β-actin was used as an internal control to verify basal level expression and equal protein loading. The abundance ratio to β-actin was calculated.

### Immunoprecipitation

Cellular extracts were prepared as described previously [35]. The obtained supernatant was mixed with protein-G beads, incubated for 2 h, and centrifuged for 2 min at 2000 rpm for pre-clearing. Then the supernatant was incubated overnight with anti-serine antibody and protein-G beads. The immunoprecipitates were collected and washed 3 times with RIPA buffer (50 mM Tris, pH7.4, 150 mM NaCl, 1% NP-40, 0.25% sodium deoxycholate, 1 mM Na_3_VO_4_, 1 mM NaF, and protease inhibitor) and finally subjected to immunoblotting analysis by Rho GTPase, ferritin, RNA polymerase, torsin-1A or LYRIC antibody.

### Construction of expression vectors

A LYRIC DNP fragment was generated from human genomic DNA using PCR. The primers used were Primer 1 (5′-TTCCCTCGACTATCCACTGCGT-3′) and Primer 2 (5′-TTCACGTGTCTCG TCTGGCTTT-3′, GenBank: AY974040.1), and the fragment was cloned into the *Bam*HI/*Xho*I site of the pcDNA3.1 vector (Amersham Biosciences) to generate the pcDNA3.1-LYRIC plasmid. Additionally, using pcDNA3.1-LYRIC plasmid as the template, a pcDNA3.1-LYRIC mutant, in which serine 568 was mutated into proline 568, was generated by the QuikChange II Site-Directed Mutagenesis Kit with LYRIC mutant primers (Primer 3, 5′-TAGCTGGGAACCTCCCAAAC-3′, and Primer 4, 5′-GTTTGGGGGATTCCCAGCTA-3′). All constructs were confirmed by restriction enzyme mapping and DNA sequencing.

### Gene transfection and stably transfected cell lines

The 6-10B cells were transfected with pcDNA3.1 (mock), pcDNA3.1-LYRIC, pcDNA3.1-LYRIC-mutant using Lipofectamine 2000 reagent (Life Technologies, Inc. Carlsbad, CA) following the manufacturer’s protocol. Stably transfected cell lines were obtained by selection for G418 resistance (400 μg/mL) as described previously [27] and further confirmed by assessing LYRIC and phos-LYRIC expression. To confirm whether DNP promotes metastasis through LYRIC phosphorylation, 6-10B-pcDNA3.1, 6-10B-LYRIC, and 6-10B-LYRIC-mutant cells were treated with DNP, and their motility and invasiveness were quantified using the in vitro Boyden chamber invasion assay.

### Bioinformatics analysis

The sub-cellular localization of these identified phosphoproteins was searched against the UniProt database and analyzed with the Gene Ontology (GO) database (http://www.geneontology.org). These identified phosphoproteins were categorized by the PANTHER (Protein Analysis through Evolutionary Relationships) system based on their biological process, molecular function, protein class, and molecular pathway (http://www.pantherdb.org). The signaling pathways of these identified phosphoproteins were mapped using the Pathway Studio program based on post-translational modifications (mainly phosphorylation) (http://www.ariadnegenomics.com/products/pathway-studio/).

### Immunohistochemistry

The metastasized nodes in the nude mice lungs were embedded, and 4-μm-thick tissue sections were made, and deparaffinized in xylene, rehydrated in a graded alcohol series, and treated with an antigen retrieval solution (10 mM/L sodium citrate buffer, pH 6.0). The sections were incubated with Lyric antibody (Biocompare, dilution 1:100) or phosho-LYRIC antibody (Abcam, dilution 1:50) overnight at 4°C. Subsequently, the sections were incubated with a biotinylated secondary antibody (Zhongshan, China), followed by incubation with an avidin–biotin complex (Zhongshan, China) following the manufacturer’s instructions. Finally, the tissue sections were incubated with 3′,3′-diaminobenzidine (Sigma-Aldrich) and with hydrogen peroxide for 2 min, and counterstained with hematoxylin for 30 s. In negative controls, the primary antibodies were replaced with normal IgG.

Under light microscopy (Olympus), the distribution of phospho-LYRIC in the nucleus and cytoplasm of the cells was rated according to a score that determined the scale of intensity of staining to the area of staining using ImageMaster software. At least 10 high-power fields were chosen randomly, and >100 cells were counted for each section.

## Results

### Analysis of SILAC labeling efficiency

The 6-10B cell line was used as a model to investigate the mechanism of DNP-mediated NPC metastasis. As a first step in our study, we assessed the incorporation efficiency of ^2^H_4_-L-lysine and ^13^C_6_^15^N_4_-L-arginine in 6-10B cells, and tested their complete incorporation in all proteins after six cell doublings. Three peptides, VEVTEFEDIK, GHYTEGAELVDSVLDVVR, and LRQPFFQK, were separated by 4 Da, 10 Da, and 14 Da, corresponding to the mass difference between the above-mentioned light and heavy isotopes. The entire signal corresponded to the heavy peptide, indicating that incorporation of ^2^H_4_-L-lysine or ^13^C_6_^15^N_4_-L-arginine was complete.

### Non-cytotoxic concentration of DNP on 6-10B cell

DNP is an important carcinogenic N-nitroso compound for NPC, and its chemical structure is shown in Figure 1A. In this study, we first determined the non-cytotoxic concentration of DNP by treating the labeled 6-10B cells with various DNP concentrations for 48 h and then subjecting the cells to an MTT assay. Compared with the controls (0.01% DMSO), the inhibitory rate of DNP on the labeled 6-10B cells was not significantly altered at 0.5–8 μM DNP (Figure 1B; p < 0.05). To confirm that 0.5–8 μM DNP was non-cytotoxic, LDH activity in the cell culture media was evaluated after DNP treatment. The data revealed that LDH activity was not significantly altered by DNP treatment in the 0.5–8 μM concentration range (Figure 1C; *p* < 0.05). This non-cytotoxic concentration range was used in all subsequent experiments.

### DNP induces the invasion and motility of 6-10B cells

The 6-10B cells exhibit lower metastasis, and were therefore used to determine whether DNP induces NPC cell metastasis. To determine whether DNP can induce the invasion and motility of the labeled 6-10B, a Matrigel-coated Boyden chamber was used to measure cell invasion, and an uncoated Boyden chamber was used to assess cell motility. After DNP treatment, the number of invaded cells dramatically increased in the Matrigel-coated Boyden chamber (Figure 2A-b) and the uncoated Boyden chamber (Figure 2A-d) as compared with the controls (Figure 2A-a, A-c). These results indicated that DNP induces 6-10B cell invasion and motility. For dose–response experiments, the cells were treated with 0, 2, 4, 6, or 8 μM DNP for 24 h and seeded into Boyden chambers, and the cells that invaded the lower chamber were then counted. The number of invading cells significantly increased after DNP treatment in a dose-dependent manner (Figure 2B-a, lanes 2 to 5 vs. lane 1; p < 0.05). The increase in cell invasion was at 421.7% with 6 μM DNP (Figure 2B-a, lane 4). A similar effect was observed in the motility of DNP-treated cells (Figure 2B-b, lanes 2 to 5 vs. lane 1; p < 0.05). Cell motility increased by 328.2% after treatment with 6 μM DNP (Figure 2B-b, lane 4). Further, the induction of metastasis by DNP was confirmed in vivo when the 6-10B cells were injected into the tail veins of BABL/c nude mice. Metastasis of 6-10B cells to the lung significantly increased after DNP treatment (Figure 2C, right vs. left panel). These results indicate that DNP can induce NPC cell motility and invasion.

**Figure 2:** **DNP-induced NPC cell metastasis in vitro *and vivo*. A**, To determine DNP-induced invasion and motility, a Matrigel-coated Boyden chamber was used to measure 6-10B cell invasion, and an uncoated chamber for measuring cell motility. The cells invading to the lower surface of Boyden chamber membrane were fixed with methanol and stained with hematoxylin and eosin. **a**, 6-10B treated with 0.01% DMSO-PBS in Matrigel-coated Boyden chamber; **b**, 6-10B cells treated with DNP (6 μM) in Matrigel-coated Boyden chamber; Scale bar, 5 μm; **c**, 6-10B cells treated with 0.01% DMSO-PBS in the uncoated chamber; **d**, 6-10B cells treated with DNP in the uncoated chamber. Scale bar, 10 μm. Arrows, The invading cells. **B**, In concentration-course assays, 6-10B cells were treated with 2, 4, 6, and 8 μM DNP for 24 h. The motility and invasion of the treated cells were analyzed. Random fields were counted to determine the number of invaded cells under a light microscope. **a**, Invasion of 6-10B cells at various concentrations; **b**, Motility of 6-10B cells at various concentrations. The results were statistically analyzed by one-way analysis of variance (ANOVA) with post-hoc Dunnett’s test (*, p < 0.05). **C**, In animal experiments, 20 nude mice were randomly divided into 2 groups with 10 mice per group. One group was injected with DNP-treated 6-10B cells in Matrigel through the tail vein (1 × 10^4^ cells/mouse). The other group was injected with untreated 6-10B cells. After 60 days, metastatic tumors nodes in the lungs were observed under the microscope (*, *p* < 0.05).

### Identification of phosphorylated proteins and their sites of modification

We employed 48-h DNP treatment for identifying DNP-regulated serine/threonine phosphorylation of proteins and their signaling components using a SILAC quantitative proteomics approach. In 3 independent experiments, more than 130 phosphopeptides were detected after manual confirmation of the MS/MS spectra by combining phosphopeptide enrichment with MS-based SILAC quantitative proteomics. All MS/MS spectra are available via the hyperlinks within Additional file 1: Table S1. To assign the phosphorylation sites precisely within a peptide, we used the PTM score to calculate the probabilities of phosphorylation at each site as previously described [32]. We were able to localize 216 phosphosites with high confidence as class I phosphorylation sites (p > 0.75). Approximately 49.6% of the phosphopeptides identified was found to be phosphorylated in a single site, and other fractions were either phosphorylated doubly (34.4%), triply (15.3%), or at more (0.8%) sites (Figure 3A). It is worth pointing out that many of these identified phosphopeptides are important signaling molecules such as protein kinases, receptors, phosphatases, and transcriptional regulators, including transcription factors and repressors (Additional file 1: Table S1).

**Figure 3:** **Characterization of phosphopeptides, phosphosites, and phosphoproteins.** The 6-10B cells with 48-h DNP treatment were used to identify DNP-regulated serine/threonine phosphorylation of proteins. To assign the phosphorylation sites precisely within a peptide, the PTM score was used to calculate the probabilities of phosphorylation at each site as described in the methods. **A**, Distribution of peptides with single, double, triple, and quadruple (including higher) phosphorylation peptides. **B**, Distribution of the Ser, Thr, and Tyr phosphosites in the DNP-regulated phosphoproteome. Phosphopeptides were categorized into class I and class II phosphosites by calculating the probabilities for phosphorylation at each site based on PTM scores. Here, only class I phosphosites (high probability) were used to analyze the distribution. **C**, Subcellular location of the phosphoproteome in vivo and GO analysis of DNP-regulated phosphoproteome. **D**, Total phosphoprotein scores of 6-10B cells with or without DNP treatment.

### Properties of phosphorylated proteins and phosphorylation sites

Figure 3B shows the distribution of identified class I phosphorylation sites, with 17 phosphotyrosine sites (2.7%), 21 phosphothreonine sites (9.58%), and 192 phosphoserine sites (87.7%). Each phosphoprotein was searched against the UniProt database (released on March 3, 2009) and analyzed using GO. Figure 3C illustrates the GO analysis for the identified phosphoproteome. The GO subcellular location information was annotated for 131 phosphoproteins. Interestingly, several cytoplasmic phosphoproteins are listed in the GO annotation (95, 72.5%) and in the UniProt database (78, 59.5%).

### Differential expression of phosphopeptides mediated by DNP

SILAC quantitative analysis of phosphopeptides was utilized to identify the DNP-mediated effects. Among the identified 131 peptides, 30 peptides were quantified, indicating significant differences in their expression between the control and DNP-treated cells. Figure 4 shows the results of the quantitative analysis of Rho GTPase protein 10 (Figure 4A) and torsin-1A protein 1 (Figure 4B) by SILAC. The data revealed 30 unique phosphopeptides containing 48 phosphorylation sites with 1.5-fold or higher changes in peak intensities in response to DNP treatment. Additional file 2: Table S2 lists these phosphopeptides with change ratios, their phosphosites and corresponding proteins, and the RSD. The comparison of the absolute values of the log2 ratios for these phosphopeptides by scatter plot analysis had a strong correlation between two biological replicates, with a Pearson coefficient of 0.874, indicating the reproducibility of these results (Figure 5A). To determine the quantitation error of phosphopeptides, DNP-regulated protein expression changes were used to determine the median H/L ratio. As shown in Figure 5B, a majority (76.9%) of the proteins was not influenced by DNP, and the SILAC ratio distribution was reasonable. Among the 30 different phosphopeptides, the phosphorylation of 48 phosphosites was inhibited by DNP, while the phosphorylation levels of only 10 were up-regulated (Additional file 2: Table S2). Moreover, the up-regulated peptides were phosphorylated at serine and tyrosine residues, but not at threonine. Serine/threonine phosphorylation sometimes attenuates the activation of signaling molecules through negative feedback [36,37]. The expression of phosphorylated peptides/proteins is probably regulated by DNP through one or more of the following methods: (1) decreasing protein expression, (2) decreasing the degree of protein phosphorylation, or (3) inducing novel phosphorylation. Among the 30 phosphoproteins, we identified 3 receptors, 1 signal adaptor, 5 protein kinases, 2 protein phosphatase regulatory subunits, 10 transcriptional regulators, and other signaling molecules as being regulated by DNP (Additional file 2: Table S2). These were the key components in the signaling pathways mediated by DNP.

**Figure 4:** **Examples of quantitative analysis by SILAC.** SILAC quantitative analysis of phosphopeptides was used to identify DNP-mediated effectors. Some peptides were quantified and showed fold differences between the control and DNP-treated cells. **A**, A representative mass spectrum showing a peptide pair (GLRDpSHpSpSEEDEASSQTDLSQTISK from Rho GTPase) with a doubly charged ion differing by 3 Da and exhibiting a H/L (of XIC) ratio of 0.35802; **B**, A representative mass spectrum a peptide pair (KFNMIPFEHRpSGGK from torsin-1A protein 1) with triply charged ions differing by 2 Da and exhibiting a H/L (of XIC) ratio of 3.2498.

**Figure 5:** **Estimation of the correlation between log 2 phosphopeptide ratios in 2 independent experiments and quantitation error of SILAC ratios of DNP-regulated proteins. A**, Two biological replicates were analyzed to compare absolute values of the log2 ratios for the phosphopeptides using scatter plot analysis. The “ratio-of-ratios” correlation between log2 phosphopeptide ratios obtained from 2 independent experiments. **B**, To determine the quantitation error of phosphopeptides, DNP-regulated protein expression changes were used to determine the median H/L ratio.

### Validation of different phosphoproteins

To verify phosphorylation levels of different proteins, the up-regulated proteins LYRIC, RNA polymerase, ferritin, and Rho GTPase were detected using phospho-serine antibody by immunoprecipitation and immunoblotting. Compared with the control, the phosphorylated forms of Rho GTPase (Figure 6A), ferritin (Figure 6B), LYRIC (Figure 6C), and RNA polymerase (Figure 6D) increased in the 6-10B cells with DNP treatment. Similarly, the decrease in the expression of phosphorylated torsin-1A protein 1 in 6-10B cells treated with DNP was also confirmed. DNP down-regulates the expression of these phosphoproteins (Figure 6E). The trends of these immunoblotting results, for all the selected proteins, were consistent with the corresponding SILAC quantitative ratios, which indicate the potential association with cancer metastasis.

**Figure 6:** **Validation of SILAC-based quantitation by immunoprecipitation and immunoblotting.** After treatment of the 6-10B cells with DNP (6 μM), cellular proteins were extracted as described in the methods. Rho-GTPase **(A)**, ferritin **(B)**, LYRIC **(C)**, RNA polymerase **(D)**, and torsin-1A protein 1 **(E)** were immunoprecipitated from the protein samples by using their corresponding antibodies, and then serine phosphorylation in the immunoprecipitated mixture was detected by immunoblotting using phospho-antibody against serine. The relative immunoblotting ratio of the phosphorylation level of every protein was normalized to its corresponding immunoprecipitated protein. IP, immunoprecipitation. IB, immunoblotting. SILAC, stable isotope labeling by amino acids in cell culture.

### DNP-mediated invasion and motility is facilitated by phospho-LYRIC expression

LYRIC, also known as metastasis adhesion protein [38,39], has been shown to promote tumor cell migration and invasion [39]. To investigate whether DNP-mediated LYRIC is involved in NPC metastasis, we first detected phospho-LYRIC expression in NPC tissues, and found that phospho-LYRIC Ser 568 is highly expressed in NPC tissues, which was expressed at higher levels in metastatic tissues than in primary site tissues (Additional file 3: Figure S1). COOH terminal-extended (amino acid 546–582) is the predominant site of regulation of nuclear localization, and its modification by ubiquitin regulates LYRIC nuclear localization [40]. Because our MS/MS data indicate that DNP mediates the phosphorylation of LYRIC at serine 568, we speculate that this phosphorylation influences NPC metastasis. To determine whether DNP-mediated LYRIC phosphorylation participates in NPC metastasis, the cells were transfected with pcDNA3.1-LYRIC. The cell motility and invasion were dramatically increased after transfection (Figure 7B, *p* < 0.05). When the cells were then transfected with pcDNA3.1-LYRIC-mutant, in which the LYRIC phosphorylation site at serine 568 was mutated (Figure 7A, lane 3 in upper panel), DNP-induced motility and invasion were considerably decreased (Figure 7B, lanes 3 and 4; Figure 7C, lanes 3 and 4). However, DNP could effectively induce cell motility (Figure 7C, lane 1 vs. 2, *p* < 0.05; Figure 7C, lane 5 vs. 6, *p* < 0.05) and invasion (Figure 7B, lanes 1 vs. 2, *p* < 0.05; Figure 7B, lanes 5 vs. 6, *p* < 0.05) when the LYRIC was not mutated. LYRIC phosphorylation at serine 568 may play an important role in DNP-mediated NPC metastasis. To confirm whether DNP has a similar effect on other NPC cells, the NPC cell line CNE1 was used to detect phospho-LYRIC, LYRIC, motility and invasion after DNP treatment. The results showed that DNP could effectively induce CNE1 motility (Figure 7D-b) and invasion (Figure 7D-c), following phosphorylation and expression of LYRIC (Figure 7D-a).

**Figure 7:** **DNP induces motility and invasion through LYRIC phosphorylation.** The 6-10B cells were transfected using pcDNA3.1, pcDNA3.1-LYRIC or pcDNA3.1-LYRICmutant, and then the stably transfected 6-10B-mock, 6-10B-LYRIC and 6-10B-LYRICmutant cell lines were obtained by selection for G418 resistance. LYRIC and phospho-LYRIC expressions were detected in these cells with or without DNP treatment **(A)**. β-actin was used as a loading control. Motility **(B)** and invasion **(C)** of 6-10B-mock, 6-10B-LYRIC, and 6-10B-LYRICmutant cells were determined in these cells. **D**, CNE1 cells were treated with DNP at 6 μM, and LYRIC and phospho-LYRIC expressions were detected using immunoblotting **(a)**, and motility **(b)** and invasion **(c)** were measured using Boyden chamber in these cell samples. Data are presented as means ± SD from 3 independent experiments. Results were analyzed using one-way ANOVA with post-hoc Dunnett’s test (*, p < 0.05).

To further determine whether DNP-mediated LYRIC phosphorylation at serine 568 is associated with NPC metastasis in vivo, phospho-LYRIC expression was detected in metastatic nodes in the nude mice lungs by immunohistochemistry. Phospho-LYRIC expression was higher in the metastatic tumors of DNP-treated mice (Figure 8A-b) than in those of the untreated control mice (Figure 8A-a). The COOH terminal of LYRIC (amino acid 546–582) is the predominant regulator of nuclear localization [40], and its phosphorylation may regulate LYRIC nuclear localization. To confirm whether DNP-mediated phospho-LYRIC regulates its nuclear localization, the phospho-LYRIC ratios of the nucleus to the cytoplasm were determined in metastatic tumor cells. The results illustrated in Figure 8B indicate that the ratio (nucleus to cytoplasm) was higher in metastatic tumors with DNP treatment than in NPC in situ from the untreated tumor. Together, our data indicate that DNP mediates LYRIC expression and phosphorylation, increases cell motility and invasion, and facilitates NPC metastasis (Figure 8C).

**Figure 8:** **Phospho-LYRIC and LYRIC expression in the metastatic tumors induced by DNP.** The metastatic tumor samples were embedded. Tissue sections of 4-μm thickness were prepared, and deparaffinized in xylene, and rehydrated in a graded alcohol series. Phospho-LYRIC and LYRIC were detected in these sections using immunohistochemistry. **A**, Paraffin sections were stained with hematoxylin and eosin as well as with antibodies against or LYRCI or phospho-LYRIC S568. **a**, **c** and **e**, The untreated 6-10B cells (NPC in situ) used as control; **b**, **d** and **f**, The DNP-treated 6-10B cells. Arrow, positive cell. Magnification, × 400. Scale bar, 5 μm. H & E, hematoxylin and eosin. **B**, Phospho-LYRIC was quantified in the nucleus and cytoplasm of metastatic tumor cells by using ImageMaster software, and phospho-LYRIC rates of nucleus to cytoplasm were calculated. **C**, Schematic illustration of DNP-induced metastasis. DNP-mediated LYRIC phosphorylation increases the motility and invasion, leading to metastasis of NPC cells.

## Discussion

In clinical settings, NPC is considered as a highly invasive and metastatic cancer. Clinical assays indicated that NPC patients with metastasis have a higher level of DNP in the serum than patients without metastasis [13].Our previous work showed that DNP is known to mediate ezrin phosphorylation and promote NPC metastasis [13]. Therefore, we speculated that DNP also induces the phosphorylation of other proteins when mediating metastasis. In the present study, we first confirmed DNP-mediated NPC metastasis, and subsequently used phosphoprotein proteomics to comprehensively identify DNP-regulated phosphoproteins and phosphosites. We found that DNP increased the expression of phosphorylated LYRIC, ferritin, Rho, and GTPase protein, and decreased the expression of phosphorylated ANKIB1 protein, dynein heavy chain 17, eukaryotic translation initiation factor 4B, triosephosphate isomerase, torsin-1A protein 1, membrane-associated progesterone receptor component 2, nuclear casein kinase, cyclin-dependent kinase substrate 1, and nucleolar RNA helicase, which are associated with protein synthesis, cellular movement, molecular transport, cell death, and signaling pathways related to cellular growth and proliferation.

Ferritins are important regulators of intracellular iron content. They are made of 24 subunits assembled to form the apoferritin shell. The protein subunits are of two types, light chain and heavy chain, which share extensive homology. Increased ferritin concentration in tumors has been recently reported in several malignancies, such as colon and breast cancers [41-43], and seminoma. Patients with NPC have higher levels of ferritin in the serum [44], and ferritin has been reported to be associated with NPC development [45]. Furthermore, high ferritin expression can enhance celluler growth and improve resistance to oxidative stress in metastatic cancer cells by interfering with their cellular antioxidant system [46]. Ferritins play important roles in chemokine receptor (CXCR)-mediated cell migration by forming a complex with CXCR4 [47]. Phospho-ferritin at serine 178 increases binding to CXCR4 and nuclear translocation. We speculate that DNP might influence NPC metastasis by regulating ferritin phosphorylation.

Initiation of transcription is a complex biological process that critically determines gene expression. Enormous efforts over the decades have revealed a set of proteins essential for this initiation by each class of eukaryotic RNA polymerases. Some of them, Drosha and Dicer, are highly expressed in NPC tissue and predict NPC prognosis [48]. For RNA polymerase I (Pol I), which is dedicated to transcription of the large rRNA precursor, 2 transcription factors have been defined in mammals. Phosphorylation at specific sites in Pol I is a prerequisite for proper transcription initiation, and phosphorylation/dephosphorylation of Pol I is one of the mechanisms by which cellular rDNA transcriptional activity could be modulated [49]. In DNP-mediated NPC metastasis, DNP might induce Pol I phosphorylation, thereby regulating DNA translocation. Activating transcription factor 7-interacting protein 1 (ATF7IP) is highly expressed in human cancers of many different tissues, suggesting that it has an important role in tumorigenesis. ATF7IP is required for the Sp1-dependent maintenance of telomerase activity in cancer cells. Hepatocyte growth factor/scatter factor (HGF/SF) is a pleiotropic cytokine/growth factor that is capable of inducing a remarkable variety of biological activities, including cellular proliferation, scattering, tubulogenesis, and invasiveness. HGF/SF can induce cyclin D1 expression in mouse melanoma cells, and this up-regulation is mediated in part by activating transcription factor-2 [50]. Rho family GTPases, including RhoA, B, C, Rac1, 2, and Cdc42, control cellular morphology and motility [51]. Many of these effects are attributed directly or indirectly to their ability to regulate the cytoskeleton. The most distinct effects of these GTPases were noted in Swiss 3 T3 cells, in which RhoA induced stress fiber formation and Rac1 induced membrane ruffling and lamellipodia, whereas Cdc42 induced spike-like filopodia [40]. In a previous study, Rho GTPase gene (*DLC1*) is inactivated by DNA methylation, and was negatively regulated in NPC carcinogenesis, whereas DLC-1 expression was detected in NPC cells after 5-aza-dC treatment [52]. In our previous work, we found that DNP activates Rho kinase and PKC, induces ezrin phosphorylation at threonine 567, increases fiber growth, and promotes motility and invasion of cells [13]. In the present study, phospho-ezrin was not detected, probably because of the incompatibility of TiO_2_ phosphopeptide enrichment or SILAC for ezrin phosphorylation at threonine. Nevertheless, DNP mediated the expression of Rho family GTPase and induced cancer metastasis. We believe that DNP also mediates NPC metastasis by increasing the expression of Rho family GTPases. LYRIC protein, also known as metastasis adhesion protein, is involved in cancer metastasis [44]. Using the evidence from two independent experiments, we suggest that DNP mediates NPC metastasis by inducing LYRIC phosphorylation at serine 568. First, DNP enhanced cell motility and invasion following higher expression of phospho-LYRIC. When the LYRIC phosphorylation site serine 568 was mutated, DNP-mediated motility and invasion was dramatically decreased. Secondly, higher levels of phospho-LYRIC were detected in DNP-induced metastatic tumors. Additionally, higher phospho-LYRIC expression at serine 568 was also detected in the NPC tissues, and it was expressed at higher levels in the metastatic tissues than in primary site tissues (Additional file 3: Figure S1). The COOH terminal of LYRIC (amino acid 546–582) is the predominant regulator of nuclear localization, and its modification by ubiquitin regulates LYRIC nuclear localization [40]. We speculate that DNP mediates the phosphorylation of LYRIC at serine 568, and regulates LYRIC nuclear localization, thereby enhancing its function and facilitate NPC metastasis. However, the function of phospho-LYRIC is not still clearly understood. Further studies are required to clarify whether LYRIC phosphorylation regulates LYRIC nuclear localization, and which kinase mediates LYRIC phosphorylation, in order to elucidate the mechanism that drives the enhanced metastasis of NPC.

## Conclusion

DNP regulates multiple signaling pathways through protein phosphorylation, including LYRIC at serine 568, and mediates NPC metastasis. These findings provide insights on the complexity and dynamics of DNP-involved metastasis, and may facilitate a better understanding of the mechanisms that favor the enhanced metastasis of NPC.

## Competing interest

The authors declare that they have no competing interest.

## Authors’ contributions

Conceived and designed the experiments: DH, FT. Performed the experiments: DH, YL, NL, ZZ, ZP, XT, GT, GY. Analyzed the data: GY, YL, NL, FT. Contributed reagents/materials/analysis tools: DH, CD, ZP, GY, FT. Wrote the paper: DH, FT. All authors read and approved the final manuscript.

## Pre-publication history

The pre-publication history for this paper can be accessed here:

http://www.biomedcentral.com/1471-2407/14/243/prepub

## Supplementary Material

Additional file 1: Table S1 DNP-regulated phosphopeptides identified using a SILAC quantitative proteomics approach. Click here for file

Additional file 2: Table S2 Different phosphopeptides mediated by DNP. Click here for file

Additional file 3: Figure S1 Phospho-LYRIC expression in the primary and metastatic tumor tissue of NPC patient. 31 primary NPC tissues were from the nasopharyngeal biopsy tissues of NPC patients, and 27 metastatic tumor tissues were from the cervical lymph metastatic node. The primary NPC and metastatic tumor samples were embedded, and 4 μm-thick tissue sections were deparaffinized in xylene, rehydrated in a graded alcohol series. Phospho-LYRIC was detected in these sections using immunohistochemistry. a, Primary NPC paraffin sections were stained with antibody against phospho-LYRIC S568; b, Metastatic tumor tissues were stained with antibody against phospho-LYRIC S568; c, Primary NPC tissues were stained with hematoxylin and eosin; d, Metastatic tumor tissues were stained with hematoxylin and eosin. Arrow, positive cells. Original magnification, × 400. Scale bar, 5μm. H & E, hematoxylin and eosin. Click here for file
